The article "The Control Index for the Construction of Sponge City in the Residential Area: A Case Study of Nanjing Jiangbei New District" was published in 2022. Journal: J Environ Public Health.

# The Control Index for the Construction of Sponge City in the Residential Area: A Case Study of Nanjing Jiangbei New District

**DOI:** 10.1155/2022/2209161

**Published:** 2022-07-14

**Authors:** Jianshi Liu, Jing Yang, Hao Zhang

**Affiliations:** ^1^School of Architecture and Urban Planning, Nanjing University, Nanjing 210000, Jiangsu, China; ^2^Nanjing Anju Construction Group Co., Ltd., Nanjing 210000, Jiangsu, China; ^3^School of Architecture, Southeast University, Nanjing 210000, Jiangsu, China; ^4^Government Service Center, People's Bank of China, Beijing 10080, China

## Abstract

The construction of sponge cities is a crucial measure for the development of an ecologically sensitive urban civilization in China, but a systematic and comprehensive construction control target has not yet been established. Considering the Nanjing Jiangbei New District as an example, this article explores how to decompose the control objectives of stormwater management in urban regions into four levels, namely, urban areas, control planning units, implementation plots, and individual technical measures, which will form the basis for the design of sponge cities. The findings of this study are expected to serve as a reference for other regions of China in the design of rainwater management systems, which form the structural backbone of the sponge cities.

## 1. Introduction

Water is one of strategic sources at a global scale [1]. With the development of mega cities and as a consequence of the massive expansion of urban construction at an unimaginable rate and scale, the urban hard ground gradually replaced the natural permeable surface of the original environment. As the area of the hardened underlying surface of the city expanded gradually, the natural water storage capacity of the surface shrank correspondingly. Consequently, during rains, the surface runoff increases sharply and flows into the stormwater drainage causing serious overload on the urban drainage system leading to waterlogging issues and causing various urban-flood related disasters. The problem of urban rainwater not only restricts the development of the cities but also threatens the safety of residents' lives and their property.

Since the 1960s, developed countries in the West have paid serious attention to urban stormwater management. Through the introduction of a series of policies and measures focused towards comprehensive management of stormwater, this has gradually become a new development trend. Through long-term practice and exploration, a set of rainwater management systems conforming to the characteristics of the country have been formed [2]. The U.S. Environmental Protection Agency proposed Best Management Practices (BMPs) in 1972 [3], combining nonengineering measures with engineering measures to control runoff pollution and total runoff, and protect the urban water environment [4]. BMP measures have been widely used in Germany, New Zealand, South Africa, and other countries and regions as well and have achieved promising results. In the 1990s, the United States put forward the concept of Low Impact Development (LID) on the basis of BMPs, which is more suitable for small-scale stormwater management [5]. Its core idea is to maintain the same hydrological characteristics before and after site development [6]. In 1994, Australia put forward the concept of Water Sensitive Urban Development (WSUD) based on studies and findings with its own unique characteristics [7]. By combining the urban water cycle process, urban planning, and landscape design with the goal of sustainable development of urban space, comprehensive water management adapted to the natural water system was realized [8]. The British government first proposed the concept of Sustainable Urban Drainage Systems (SUDS) in 1961 [9]. Through planning and design, various urban drainage systems were considered as a whole and sustainable development concepts and measures were introduced to optimize the overall hydrological environment [10]. Although the Western countries have their own emphasis on the concept and construction mode of stormwater management, their extensive practice and application provides experience and serves as a reference for the construction of urban stormwater management in China.

The article "The Control Index for the Construction of Sponge City in the Residential Area: A Case Study of Nanjing Jiangbei New District" was published in 2022. Journal: J Environ Public Health.

Over the past 30 years, various reforms and the opening up of the economy in China have spurred urban development and the urbanization rate has continued to grow unabatedly. In 2016, China's urbanization rate reached 57.35% [11] and continues to maintain a rapid development momentum; by 2020, it was expected to exceed 60% [12]. In China, the process of urbanization along with the scale of expansion of the cities has brought sustained and rapid development to the society, while simultaneously it has also led to the continuous hardening of the land and the extent of impervious areas in cities has rapidly expanded. About 90% of the urban rainfall forms run off, and this has resulted in a series of environmental problems such as urban waterlogging and water pollution: 360 cities in China suffered waterlogging in the three-year period from 2012 to 2015. Waterlogging happens every time it rains and it has become one of the major urban disasters in China. As such, contemporary China is facing various water resource crises such as water shortages, water pollution, and floods [13].

To alleviate the aforementioned problems, China has put forward the concept of sponge city construction. In 2013, General Secretary Xi Jinping proposed the concept of sponge city at the Central Urbanization Work Conference. Subsequently, in 2014, the Ministry of Housing and Urban-Rural Development issued the “Technical Guidelines for Sponge City Construction (Trial),” which established the basic principles, content, requirements, and methods of sponge city construction. In the work report of the two sessions in 2017, Premier Li Keqiang emphasized the importance of coordinating the construction above and below the ground in urban areas simultaneously, which typically includes the construction of comprehensive underground pipe corridors of more than 2,000 kilometers [14]. The three-year action plan to promote the construction of sponge cities to eliminate water logging in key areas and make the cities more attractive and function better was initiated by him [12]. The development direction of sponge cities has been clearly defined. The construction of the sponge city has not been limited to pilot cities alone because it has become a functional necessity that all cities must pay attention to during initial development itself.

The article "The Control Index for the Construction of Sponge City in the Residential Area: A Case Study of Nanjing Jiangbei New District" was published in 2022. Journal: J Environ Public Health.

Compared with the traditional “quick drain” urban drainage method, the sponge city has good “elasticity” like a sponge. It adopts the effective combination of green ecological methods and gray infrastructure such as seepage, retention, storage, purification, use, and drainage. The sponge city infrastructure absorbs the water during rain and releases it when needed like a sponge: to “breathe in and out” comfortably, recycle rainwater, and realize a virtuous cycle of the urban water environment. The construction of the sponge city covers three aspects: the first is the protection of the original urban ecosystem, the second is ecological reparation and restoration, and the third is low-impact development [15]. On the one hand, the sponge city enhances a city's ability to adapt to heavy rains, while on the other it uses rainwater to restore the wetland system to create basic ecological service facilities with multiple ecological service functions [6]. The “sponge body” of the sponge city includes not only the city's rivers and lakes but also the permeable paving, green roofs, green spaces, rain gardens, and other supporting facilities in the residential area.

As residential areas account for half of the total urban construction [16], they cover the widest surface area and generate the most rainwater runoff and thus play a vital role in solving the urban rainwater problem. Prioritizing research on the sponge city strategy for residential areas is of practical significance to China's promotion of sponge city construction. The construction of sponge settlements is an important measure to implement the construction of sponge cities, and it is also a strong guarantee for the restoration of the urban ecological environment. Therefore, the construction of sponge settlements is imperative.

The article "The Control Index for the Construction of Sponge City in the Residential Area: A Case Study of Nanjing Jiangbei New District" was published in 2022. Journal: J Environ Public Health.

## 2. The Status and Problems of China's Sponge Settlement Construction

Long before the concept of sponge city was put forward, China had already tried green ecological technology in residential areas. In 2004, the Shenzhen Guangming New District took the lead in introducing the concept of low-impact development in the country and achieved initial results in the low-impact development of rainwater utilization, forming a certain demonstration effect [17]. In 2015, the Ministry of Construction, the Ministry of Finance, and the Ministry of Water Resources launched the first batch of 16 pilot sponge cities: another 14 cities were added in 2016 for which the central government provided special fund subsidies. The launch of the sponge city pilot has greatly promoted the concept of sponge city in China and the creation of sponge cities has begun to take shape.

Although China has issued the “Technical Guidelines for Sponge City Construction” and the drainage specifications for rainwater utilization at the national level, there are still relatively few studies, and practices on the meso-micro-scale controlled detailed planning level for urban rainwater management goals. The planning system for sponge cities has not yet been established, and there is a lack of hierarchical rainwater utilization norms [18]. The control indicators of traditional control regulations, such as the building density and floor area ratio, are mainly based on land development control [18]. There is a lack of control indicators related to hydrological environment and urban stormwater management infrastructure, and those that distinguish between different land use [19]. Therefore, it is difficult to control the actual plots within the scope of the control regulations. Clearly defining and proposing targeted measures cannot guarantee the realization of the construction goals of sponge settlements. It is a known fact that the geographical area of a whole city is divided into urban plots, blocks, and large divisions. This paper takes the small watershed unit with an independent and completely natural hydrological ecosystem as the regional scale and basic unit of hydrological management. Furthermore, it takes the aforementioned basic unit and effectively connects with the urban space scale, forming the four planning levels of the whole city, planning unit, implementation of land parcels, and land parcel sponge measures to quantify and determine the sponge settlement control indicators. This arrangement makes each hydrological process complete and independent, and forms a hierarchical rainwater management indicator system for sponge settlements.

The article "The Control Index for the Construction of Sponge City in the Residential Area: A Case Study of Nanjing Jiangbei New District" was published in 2022. Journal: J Environ Public Health.

## 3. Research Methodology

### 3.1. Case Study Approach

A case study approach was adopted in this research in order to develop a framework for sponge settlements that will be tested in Nanjing Jiangbei New District. The case study approach is most appropriate for “How” and “Why” type of research questions. As this research aims to define how to control sponge settlements, it is appropriate to use the case study method.

### 3.2. Site Selection

Nanjing Jiangbei New District is located to the north of the Yangtze River in Nanjing, with a total area of 2,451 square kilometers. It is an important node for the Yangtze River Delta for driving the development of the middle and upper reaches of the Yangtze River (Figure 1). In June 2015, Nanjing Jiangbei New District became the 13th national-level new district in the country [20], and its development model has a demonstrative effect. In 2016, the Nanjing Municipal Government issued the “Implementation Opinions on Promoting the Construction of Sponge Cities,” establishing Jiangbei New District as a pilot project for the construction of sponge cities, thus providing an opportunity for Jiangbei New District to take a new path to urbanization and explore the construction of sponge settlements.

### 3.3. Data Collection

This paper uses Nanjing Jiangbei New District as the research area to analyze the total annual runoff index and decompose the indicators into various plots, and finally realize the decomposition of the total annual runoff index. The research process is shown in Figure 2.

## 4. Establishment and Decomposition of Control Indicators for Sponge Settlements

### 4.1. Control Target

The hydrological index system for urban stormwater management in the United States has established the following indices according to the level, namely, the infiltration control index, nonpoint source pollution control index, river erosion control index, small-scale flood control index, and extreme flood control index. The first three aim to control the total amount of runoff and focus on protecting the water environment, whereas the latter two indicators aim to control the peak runoff and reduce flood disasters in cities and downstream areas [21]. Currently, a similar hydrological control index system is applied in many other regions in different forms, such as New York [22], Washington DC [3], and other areas of the United States as well as in many cities of Australia [23]. They serve as significant references for the establishment of control indices for China's rainwater management system.

The article "The Control Index for the Construction of Sponge City in the Residential Area: A Case Study of Nanjing Jiangbei New District" was published in 2022. Journal: J Environ Public Health.

In the “Technical Guidelines for Sponge City Construction” promulgated by the Ministry of Housing and Urban-Rural Development of the People's Republic of China, the planning and control objectives for constructing a low-impact development rainwater system include total runoff control, runoff peak control, runoff pollution control, rainwater utilization, etc. The total runoff control is the primary control goal because other goals can be achieved by controlling the total volume of runoff. The decomposition of the 12-year total runoff index is an important step in the implementation of the “Technical Guidelines for Sponge City Construction” and an important guarantee for the comprehensive and orderly development of sponge settlements.

In order to decompose the total annual runoff target, it is necessary to quantify the construction control indicators of sponge settlements at the four planning levels of the city, region, control unit, and implementation land in accordance with the intensity of urban construction development and surface hydrological characteristics. To achieve the goal of constructing the sponge cities, the value of the control index needs to be determined in the sponge city construction plan at each of the four levels, i.e., the city master plan (city or regional index), planning unit master plan (plan unit index), detailed control plan (implementation plot index), and constructive detailed plan (individual control index for sponge measures). The indices of the next level must meet the weighted average of the indices of the previous level. The focus is on targeted index research and decomposition of the planning unit index and the implementation land index for the urbanized residential areas. Through four-level planning and targeted index decomposition, quantitative indicators are reasonably implemented in specific plots to guide the sponge construction of residential areas.

### 4.2. Decomposition of Total Annual Runoff Indicators

#### 4.2.1. Overall Plan

According to the “Technical Guidelines for Sponge City Construction,” through statistical analysis of the average daily rainfall data of nearly 200 cities in China over the past 30 years (1983–2012), mainland China is roughly divided into five regions according to the relationship between the total annual runoff control rate and the corresponding design rainfall value. The range of the total annual runoff control rate *α* in each region is: District I: 5% *α* ≤ 90%, District II: 80% *α* ≤ 85%, District III: 75% *α* ≤ 85%, District IV: 70% *α* ≤ 85%, and District V: 60% *α* ≤ 85% (Figure 2) [15].

The article "The Control Index for the Construction of Sponge City in the Residential Area: A Case Study of Nanjing Jiangbei New District" was published in 2022. Journal: J Environ Public Health.

As shown in Figure 3, Nanjing belongs to Zone III in the total annual runoff control zone on the mainland, and the annual runoff vacancy rate ranges from 75 to 85%. Jiangbei New District is a newly constructed urban area in Nanjing with good natural hydrological conditions. It also belongs to the pilot area of the sponge city in Nanjing. The target for the total annual runoff control rate can be appropriately increased. Through monitoring the effect of the built sponge residential area (Nanjing Dingjiazhuang security housing area), it was comprehensively determined that the lower limit of the total annual runoff of the sponge city in the Jiangbei New District should be set to 80%, corresponding to the control design rainfall of 29.7 mm [15].

#### 4.2.2. Overall Planning of the Planning Unit

The spatial planning of water areas should take the relatively independent, complete, and closed natural hydrological ecosystem as the planning unit [24]. At the level of regional planning, the current small watershed unit needs to be taken as the regional scale for decomposing the total annual runoff index of the city. By ensuring the integrity and closure of the regional hydrological process while simultaneously connecting with the urban blocks, the natural ecosystem and urban land can be effectively integrated. To ensure that the small watershed unit is used as the scale of rain and flood management, when dividing the urban unit it should overlap with the small watershed unit as much as possible. The total annual runoff control index of the planning unit can be expressed as follows:

(1) $$\begin{array}{c} p=p_{0}+p_{1}, \end{array}$$

where *p* is the total annual runoff control rate of the planning unit, *p*_0_ is the total annual runoff control rate of the city or region where the planning unit is located, and *p*_1_ is the sponge city construction suitability adjustment coefficient of the planning unit.

After dividing the stormwater management units into small watershed units, it is necessary to evaluate the sponge city construction suitability of each stormwater management unit and determine the sponge city construction suitability adjustment coefficient of each management unit *p*_1_. To meet the requirements of socioeconomic value and ecological value while extracting urban spatial elements, this paper uses three evaluation factors: population density factor, spatial integration factor, and green space system factor to evaluate the site suitability of each stormwater management unit. In the article, “Study on Location Selection of Sponge Sites in Changchun City Based on Sensitivity and Significance Analysis,” the population density factor, spatial integration factor, and green space system factor of the sponge city study area are scored from 0 to 4. Through a combination of the expert scoring method and Yaahp, the analytic hierarchy process software, the weights of the population density, spatial integration, and urban blue-green system are determined to be 0.5695, 0.3331, and 0.0974, respectively. The three suitability influencing factors are weighted and averaged to obtain a comprehensive evaluation of the suitability of sponge cities in the study area. Using the natural discontinuity classification method to take the range of 0.00∼0.38∼1.29∼2.04∼2.76∼4.00 as the comprehensive suitability classification standard, the construction of sponge cities in the study area is divided into five types: unsuitable land, less suitable land, suitable land, more suitable land, and the most suitable land [25]. Among them, the sponge city construction suitability adjustment coefficient *p*_1_ of suitable land is taken as 0; the unsuitable land and less suitable land should be moderately reduced according to the hydrogeology of the area, the actual situation of urban construction, and the overall goal of regional sponge city construction. The most suitable land should be appropriately increased according to the hydrogeology of the region, the actual situation of urban construction, and the overall goal of regional sponge city construction to achieve regional self-balance of annual runoff control and rainwater utilization.

The article "The Control Index for the Construction of Sponge City in the Residential Area: A Case Study of Nanjing Jiangbei New District" was published in 2022. Journal: J Environ Public Health.

On the basis of the total annual runoff control target in the Nanjing Jiangbei New District, the small watershed units are divided based on the administrative divisions and the river basin divisions (Figure 4). The sponge city construction suitability evaluation for each planning unit is carried out (Figure 5), and the evaluation maps of the population density factor (Figure 6), spatial integration factor (Figure 7), and green space system factor (Figure 8) of each planning area are obtained. Through the weighted average of the three suitability influencing factors, the comprehensive evaluation of the sponge city construction suitability of each planning unit in Jiangbei New District is obtained (Figure 9). The corresponding adjustment coefficient p1 of the sponge city construction suitability of the planning unit is determined according to Table 1, and the total annual runoff control target of each planning unit is determined. For example, the population density factor of the d010 plot in the central area of Jiangbei New District is 1, the spatial integration factor is 3, the green space system factor is 2, and the weighted average comprehensive evaluation of the suitability of sponge city construction is 1.7636. The results lead to the conclusion that it is suitable land for sponge city construction. The adjustment coefficient*p*_1_ of the sponge city construction suitability of the planning unit is 0; therefore, the total runoff control rate of d010 in Jiangbei New District is

(2) $$\begin{array}{c} p=p_{0}+p_{1}=80\%+0=80\%. \end{array}$$

The corresponding design rainfall is 29.7 mm.

The article "The Control Index for the Construction of Sponge City in the Residential Area: A Case Study of Nanjing Jiangbei New District" was published in 2022. Journal: J Environ Public Health.

#### 4.2.3. Controlled Detailed Planning

The total annual runoff control target of the planning unit in the overall plan of the planning unit is decomposed, and the total annual runoff control target of each residential land in the planning unit is calculated (Figure 10).

(1) The permeable paving rate and green roof rate of the planning unit is proposed based on the actual situation of the planning unit and the existing empirical data to determine the proportion of various types of land area. The runoff coefficients of different types of underlying surfaces need to be determined based on the actual measured data. If there is no actual measured data, then the value presented in Table 2 could be considered for the calculations. The comprehensive surface runoff coefficient is calculated according to the weighted average of the land types:
  (3) $$\begin{array}{c} \varphi =\frac{\sum Fi\varphi i}{F}, \end{array}$$
where *φ* is the comprehensive surface runoff coefficient, F is the planning area (m^2^), Fi is the area for the various land types in the planning unit (m2), and *φ*_*i*_ is the runoff coefficient of various land types.
(2) Rainfall in the planning unit is controlled through infiltration and green rainwater infrastructure. The total rainfall in the planning unit is expressed as
  (4) $$\begin{array}{c} V=\frac{HF}{1000}, \end{array}$$
where *V* is the total rainfall (m^3^), H is the designed rainfall (mm), and F is the planning area (m^2^).
(3) The amount of rainfall control achieved through infiltration is expressed as
  (5) $$\begin{array}{c} V_{1}=V\times \left(1-\varphi \right), \end{array}$$
where *V*_1_ is the infiltration rainfall control amount (m^3^); *V* is the total rainfall (m^3^); and *φ* is the comprehensive surface runoff coefficient.
(4) The amount of rainfall control achieved through the green rainwater infrastructure (*V*_2_=*V* − *V*_1_) is mainly controlled by the rainwater storage and retention facilities.
  (i) Rainwater storage: the rainwater regulation and storage volume *V*_*a*_ is determined according to the water area of the planning unit with the function of rainwater regulation and storage and the regulation depth reserved for rainwater regulation and storage.
  (ii) Rainwater retention: according to the actual situation of the planning unit and the existing empirical data, the rate of sinking green space and the depth of sinking green ground of the planning unit are proposed (the sinking depth should be determined according to the actual situation of the project, and it can be located at 0.1 m when there is no measured data), and the volume of rainwater storage *V*_b_ in the sunken green space can be determined.
  (iii) In addition, it is necessary to build rainwater storage facilities and the rainwater storage capacity *V*_c_ = V_2_—*V*_a_—*V*_b_, then the standard for rainwater storage facilities for every 10,000 square meters of hardened area is
    (6) $$\begin{array}{c} V_{m}=\frac{V_{c}}{F_{m}}, \end{array}$$
where *V*_*m*_ is the rainwater regulation and storage capacity of rainwater regulation and storage facilities per 10,000 square meters of hardened area (m^3^/hm^2^), *V*_*c*_ is the rainwater regulation and storage capacity (m^3^), and *F*_*m*_is the hardened area of the planning unit construction project (hm^2^).
*Note*. Hardened area: in a residential area project, the hardened area refers to the hardened area of the roof, which is calculated according to the projected area of the roof (excluding the greened roof). For nonresidential projects, the hardened area includes the hardened area of roofs, roads, squares, courtyards, etc., within the scope of construction land. The specific calculation method is “hardened area = construction land area—green area (including green roof)—permeable pavement land area.” (Nanjing City Rainwater Comprehensive Utilization Technical Guidelines (Trial))
(5) Total annual runoff control rate of residential land
  (i) The comprehensive surface runoff coefficient of residential land is determined according to the proportion of various types of residential land area, the rate of permeable paving, and the green roof of the planning unit:
    (7) $$\begin{array}{c} \varphi_{r}=\frac{\left(\sum F_{j}\varphi_{j}\right)}{F_{r}}, \end{array}$$
  where *φ*_*r*_ is the comprehensive surface runoff coefficient of residential land, *F*_*r*_ is the total planned area of residential land (m^2^), *F*_*j*_ is the residential land area of various land types (m2), and *φ*_*j*_ is the the runoff coefficient of various land types that are determined based on the measured data. If there is no measured data, the value is obtained according to Table 3.
  (ii) The amount of rainfall control achieved by the green rainwater infrastructure on residential land is expressed as
    (8) $$\begin{array}{c} V_{r2}=V_{ra}+V_{rb}+V_{m}\cdot F_{m}, \end{array}$$
  where *V*_*r*2_ is the amount of rainfall control achieved by the green rainwater infrastructure on residential land (m3); *V*_*ra*_ is the water storage capacity of rainwater (m3); *V*_*rb*_ is the rainfall storage capacity of sunken green space (m3); *V*_*m*_ is the rainwater regulation and storage capacity of rainwater regulation and storage facilities per 10,000 square meters of hardened area (m^3^/hm^2^); and *F*_*rm*_ is the hardened area of the residential land construction project (hm^2^).
  (iii) Design rainfall for residential land is expressed as
    (9) $$\begin{array}{c} H_{r}=\left(\frac{1000V_{r2}}{\varphi_{r}\cdot F_{r}}\right), \end{array}$$
  where *H*_*r*_ is the design rainfall for residential land (mm), *V*_*r*2_ is the volume of rainfall control achieved by the green rainwater infrastructure on residential land (m^3^), *φ*_*r*_ is the comprehensive surface runoff coefficient of residential land, and Fr is the total planned area of residential land (m^2^).
  (iv) According to the design rainfall,
  *H*_*r*_ value of the residential land, the designed rainfall is checked corresponding to the total annual runoff control rate of local cities and the total annual runoff control target of residential land is determined.

Taking the d010 plot in the central area of Jiangbei New District as an example, the annual runoff total control target in the detailed regulatory planning is decomposed, and the annual runoff total control target for residential land in the d010 plot is calculated.

(i) Because the “Technical Guide for Sponge City Construction” does not have unified requirements for indicators such as the permeable pavement rate and green roof rate, the selection of d010 plot indicators has been done with reference to “rainwater control and utilization engineering design specifications.” The empirical data available for existing projects at home and abroad are as follows:
Permeable paving rate of this unit ≥70%, Green roof rate of this unit ≥30%, and Concave green area rate of this unit ≥10%.
(ii) The proportions of various types of land in the d010 plot are calculated (Figure 11). The comprehensive surface runoff coefficient of the d010 block is obtained as *φ* = 0.443 by classifying and sorting based on residential land (including green roof construction land, hardened roof construction land), square road land (including permeable paving and impervious paving), green space, public municipal land, and water areas (Table 3) [10].
(iii) Total rainfall in d010 block
  (10) $$\begin{array}{c} V=\left(\frac{HF}{1000}\right)=483272m^{3}, \end{array}$$
where H is the designed rainfall, 29.7 mm, and F is the planning area, 1627.18 × 10^4^ m^2^
(iv) The volume of rainfall control achieved by infiltration in the d010 block
  (11) $$\begin{array}{c} V_{1}=V\times \left(1-\varphi \right)=269183m^{3}, \end{array}$$
where *V* is the total rainfall, 483272 m^3^, and *φ* is the comprehensive surface runoff coefficient, 0.443.
(v) The volume of rainfall control achieved by the green rainwater infrastructure in the d010 plot is *V*2=*V* − *V*1=214089*m*^3^; the green area of the d010 block accounts for 36.67% of the total area and the concave green area F′ = *F* × 0.3667 × 0.1 = 596687 m2, calculated according to the concave green rate of 10%. Assuming the depth of the concave green underground as 0.1 m, the rainfall regulation and storage of the concave green space is *V*_*b*_ = *F*' × 0.1 = 59669 m3. The d010 block needs to be equipped with rainwater regulation and storage facilities; the rainwater regulation and storage volume is *V*_*c*_=*V*_2_ − *V*_*b*_=154420*m*^3^. The construction standard of the rainwater regulation and storage facilities per 10,000 square meters of hardened area in the d010 plot is
  (12) $$\begin{array}{c} V_{m}=\left(\frac{V_{c}}{F_{m}}\right)=298\left(\frac{m^{2}}{hm^{2}}\right), \end{array}$$
where *V*_*c*_ is the rainwater regulation and storage capacity with rainwater regulation and storage facilities, 154420 m^3^, and *F*_*m*_ is the hardened area of the planning unit construction project, 517.91 hm^2^.
(vi) According to the proportion of the land area of various land types, the permeable paving rate, and green roof rate of the residential land in the d010 block in the detailed regulatory planning, the comprehensive surface runoff coefficient *φ* of the residential land in the d010 block is determined to be 0.386, as shown in Table 4.

 The amount of rainwater regulation and storage per hectare of residential submerged green space in d010 block is *V*_*b*_ = 10000 *m*^2^ × 0.3 × 0.1 × 0.1 *m* = 30 m^3^, then the amount of rainfall control achieved by the green rainwater infrastructure per hectare of residential land is

(13) $$\begin{array}{c} V_{r2}=V_{rb}+V_{m}\cdot F_{m}=82\cdot 15m^{3}, \end{array}$$

where *V*_*rb*_ is the rainwater regulation and storage capacity per hectare of residential underground sunken green space, 30 m^3^. *V*_*m*_ is the rainwater regulation and storage capacity of rainwater regulation and storage facilities per 10,000 square meters of hardened area, 298 m^3^/hm^2^, and F_rm_ is the hardened area of the construction project per hectare of residential land, 0.175 hm^2^.

(i) Designed rainfall of residential land in d010 block
  (14) $$\begin{array}{c} H_{r}=\left(\frac{\left(1000V_{r2}\right)}{\left(\varphi_{r}F_{r}\right)}\right)=21.3mm, \end{array}$$
where *V*_r2_ is the controlled amount of rainfall achieved by green rainwater infrastructure per hectare of residential land, 82.15 m^3^. *φ*_*r*_ is the comprehensive surface runoff coefficient of residential land, 0.386, and *F*_r_ is the planning area per hectare of residential land, 10000 m^2^.
(ii) According to Table 5 and Figure 12, the total annual runoff control rate of residential land in the d010 block is 71%.
To achieve the overall target of 80% of the total annual runoff control rate of the d010 plot, the lower limit of the annual runoff control rate of the residential land in the d010 block is 71%. Compared with the overall target of 80% annual runoff control rate of the planning unit, the annual runoff control target of residential land in the d010 plot can be moderately reduced.

The article "The Control Index for the Construction of Sponge City in the Residential Area: A Case Study of Nanjing Jiangbei New District" was published in 2022. Journal: J Environ Public Health.

#### 4.2.4. Constructive Detailed Planning

The total annual runoff control target for the residential land in each planning unit and the construction plot is determined according to the actual plot size, hydrogeology, flood control and drainage system, floor area ratio, green space ratio, building density and development cost, etc. The total annual runoff control target of the sponge city on the construction site is determined, and a systematic plan for the construction of the sponge city on the plot is proposed as per the target. The proportion of various technical means in the control index of the sponge city is clarified, and the low-impact development facilities are rationally arranged.

Subsequently, the individual indices of the low-impact development index of the residential area of the planning unit are determined. Because the “Technical Guide for Sponge City Construction” does not have unified requirements for indicators such as permeable pavement rate and green roof rate, the selection of settlement planning indicators is done mainly with reference to the relevant current national, local standards and regulations, the empirical data, and cost considerations of existing projects at home and abroad that assign values to low-impact development indicators as well.

Table 5 shows the relevant standards and norms currently applicable for the country, Jiangsu Province, and Nanjing City. The individual indices for the low-impact development of the residential land in the d010 block have been determined with reference to the relevant indicators in Table 5, the experience of existing projects at home and abroad, and in combination with the actual development conditions of the residential area of the d010 block in Jiangbei New District: details of the individual indices are presented in Table 6. As shown in Table 6, three major control indices are defined in regulations, i.e., permeable area ratio, sunken green space, and regulation and storage facilities. In addition, requirements have been set for low-impact development for following four components: high-end residential area, ordinary residential area, guaranteed housing, and municipal roads shown in Table 7.

The article "The Control Index for the Construction of Sponge City in the Residential Area: A Case Study of Nanjing Jiangbei New District" was published in 2022. Journal: J Environ Public Health.

## 5. The Technical Selection of Sponge City

The low-impact development technology of the sponge city can be divided into several categories, such as infiltration, storage, regulation, transfer, pollution interception, and purification, and each category contains different low-impact development measures. The main low-impact development measures, their advantages, and disadvantages are shown in Table 8.

In the “Technical Guidelines for Sponge City Construction,” the facility functions of different low-impact development measures are compared, as reproduced in Table 9 [15].

The spatial conditions and hydrological characteristics of the residential areas are taken into consideration comprehensively, including the economics, applicability, and landscape effects of various low-impact development facilities. The low-impact facilities suitable for residential sponge construction are permeable brick paving, green roof, sunken green spaces, biological retention facilities, seepage ponds, seepage wells, wet ponds, rainwater wetlands, rainwater tanks, regulating ponds, grassed swales, seepage pipes/canals, vegetation buffer belts, initial rainwater retention facilities, etc.

## 6. Conclusions

China's sponge city construction not only includes technical measures with low-impact development concepts but also protects the original urban ecosystem from a macro perspective and prevents flooding due to urban rainwater from occurring on multiple scales, i.e., in regions, cities, and blocks.

The core idea of the sponge city technology is to plan and implement ecological rainwater facilities of different scales and at different planning stages to meet goals such as runoff reduction and forming a complete stormwater management network system. As residential areas account for half of the entire city's construction, implementation of sponge city construction plays a vital role in solving the urban rainwater flooding problem. This study combines the salient points of China's sponge city construction policy initiative with the characteristics of China's residential areas to determine the actual total runoff control goals. In particular, an effective approach was explored to decompose the control objectives of stormwater management in urban regions into four levels, i.e., urban areas, control planning units, implementation plots, and individual technical measures, forming the basis for the design of sponge cities. It is revealed in this study that achievement of the construction control targets at all levels is of critical significance for gaining the entire range of environmental benefits of the sponge city construction and coordinating China's rain and flood management system at all levels. Meanwhile, this research provides an empirical reference for the decomposition of sponge city construction control goals for residential areas in other regions.

The article "The Control Index for the Construction of Sponge City in the Residential Area: A Case Study of Nanjing Jiangbei New District" was published in 2022. Journal: J Environ Public Health.

The main limitation associated with this study belongs to the nature of single case study. The overall achievement and effectiveness of measures proposed in this study could be tested in other projects.

## Figures and Tables

**Figure 1:** Location of nanjing jiangbei new district.

**Figure 2:** Research process.

**Figure 3:** The zoning map of the total annual runoff control rate in mainland China.

**Figure 4:** Water system distribution map of Nanjing Jiangbei New District.

**Figure 5:** Division of rain and flood management units in Nanjing Jiangbei New District.

**Figure 6:** Evaluation of population density factors in Nanjing Jiangbei New District.

**Figure 7:** Evaluation map of spatial integration factors in Nanjing Jiangbei New District.

**Figure 8:** Evaluation of green space system factors in Nanjing Jiangbei New District.

**Figure 9:** Comprehensive evaluation of the suitability of sponge city construction in Nanjing Jiangbei New District.

**Figure 10:** The technical route for the decomposition of the total annual runoff control target of the planning unit.

**Figure 11:** The urban construction land plan of block d010 in the central area of Nanjing Jiangbei New District.

**Figure 12:** The total annual runoff control rate in Nanjing City corresponded to the design rainfall.

**Table 1:** Sponge city construction suitability adjustment coefficient *p*_1_ in the planning unit of Jiangbei New District.

Suitability of sponge city construction	Unsuitable	Less suitable	Suitable	More suitable (%)	Most suitable (%)
Suitability adjustment factor *p*_1_	−10%	−5%	0	5	10

**Table 2:** Runoff coefficient of each land type [15].

Land type		Runoff coefficient
Residential	Green roof	0.4
	Hardened roof	0.85
Road square	Permeable	0.15
	Impermeable	0.85
Green space		0.15
Public municipal		0.85
Waters		1

**Table 3:** Estimation of comprehensive surface runoff coefficient of d010 plot.

Land type		Percentage	Runoff coefficient
Residential	Green roof	4.79	0.4
	Hardened roof	11.18	0.85
Road square	Permeable	19.5	0.15
	Impermeable	21.58	0.85
Green space		36.67	0.15
Public municipal		1.38	0.85
Waters		4.91	1
Comprehensive surface runoff coefficient		0.443	

**Table 4:** Estimation of comprehensive surface runoff coefficient of residential land in d010 plot.

Land type		Percentage	Runoff coefficient
Residential	Green roof	7.5	0.4
	Hardened roof	17.5	0.85
Road square	Permeable	31.5	0.15
	Impermeable	13.5	0.85
Green space		30	0.15
Comprehensive surface runoff coefficient		0.386	

The article "The Control Index for the Construction of Sponge City in the Residential Area: A Case Study of Nanjing Jiangbei New District" was published in 2022. Journal: J Environ Public Health.

**Table 5:** The total annual runoff control rate corresponding to the design rainfall in Nanjing.

Annual runoff control rate	35%	40%	45%	50%	55%	60%	65%	70%	75%	80%	85%	90%
Designed rainfall (mm)	6.2	7.5	9.0	10.7	12.6	14.8	17.4	20.6	24.8	29.8	36.8	48.4

*Note.* The data are from China Meteorological Administration 1981–2015.

**Table 6:** Single index requirements for low-impact development of residential land in d010 block.

Single control index		Notice of the General Office of the State Council on doing a good job in the construction of urban drainage and prevention facilities. State Office issued (2013) No. 23	“Technical Specification for Rainwater Utilization Engineering in Buildings and Residential Areas”	“Outdoor Drainage Design Plan” (GB 50014-2006)	Notice of the General Office of the Provincial Government on implementing the Notice of the General Office of the State Council on doing a good job in the construction of urban drainage and waterlogging prevention facilities Suzhou Provincial Government Office issued (2013) No. 88	Notice on issuing “Technical Guidelines for Comprehensive Utilization of Rainwater in Nanjing City (Implementation)” Nanjing Construction and Environment Agency (Implementation) Nanjing (2014) No. 612	Implementation opinions on promoting the construction of sponge city (submission for examination) Municipal Construction Committee

Permeable area ratio	No less than 40%	Among the hardened ground in the newly built urban area, the percentage of permeable ground area should not be less than 40%	Permeable ground should be used on hard ground and squares where pedestrians and nonmotor vehicles pass	Among the hardened ground in the newly built urban area, the percentage of permeable ground area should not be less than 40%	Among the hardened ground in the newly built urban area, the percentage of permeable ground area should not be less than 40%	—	Residential area: in the hardened ground, the permeability shall not be less than 40%; Road: the permeable paving rate of the newly built sidewalk is 50%, and the rebuilding rate is 30%; Park: Pedestrian system, parking lot, and other facilities adopt permeable pavement. The permeable pavement rate of new parks should not be less than 50%

Sunken green space	No less than 10%	—	The road surface in the residential section should be 50–100 mm higher than the roadside green space	The elevation of the green space should be 5–25 cm lower than the elevation of the surrounding ground to form a recessed green space	—	For all construction projects that involve the requirements of the green space rate index, 30% of the green space should be used as a recessed green space for retaining rainwater	For all construction projects that involve the requirements of the green space rate index, at least 10% of the green space should be used as recessed green space for retaining rainwater, and the green space in urban parks should not be less than 30% recessed

Regulation and storage facilities	No less than 100 m^3^/ha	—	—	—	Urban construction should pay attention to rainwater collection and utilization, with a construction standard of 100 m^3^/ha	For new buildings with a planned construction land area of more than 20,000 square meters, a rainwater collection and utilization system must be built; the standard is 100 m^3^/10,000 m^2^	The planned construction land of 20,000 square meters shall be equipped with a rainwater collection and utilization system

The article "The Control Index for the Construction of Sponge City in the Residential Area: A Case Study of Nanjing Jiangbei New District" was published in 2022. Journal: J Environ Public Health.

**Table 7:** Single index requirements for low-impact development of residential land in d010 plot.

Control index	High-end residential area	Ordinary residential area, guaranteed housing	Municipal roads
Subsidence green rate	≥ 15%	≥ 10%	≥ 30%
Green roof rate	20%–50%	—	—
Permeable pavement rate	≥ 90%	≥ 70%	≥ 90%
Regulation and storage facilities	Every 10,000 square meters of the hardened area is equipped with a rainwater storage facility of not less than 300 m^3^		—

**Table 8:** Advantages and disadvantages of main low-impact development measures.

Technical measures	Advantages	Disadvantages
Permeable paving	Wide application area, convenient construction, can replenish groundwater and have a certain peak flow reduction and rainwater purification effect	Easy to block, cold areas are at risk of being destroyed by freezing and thawing
Green roof	Can effectively reduce the total amount of roof runoff and runoff pollution load	There are strict requirements on roof load, waterproofing, slope, space conditions, etc.
Sunken green space	Wide application area, its construction cost and maintenance cost are low	Easily affected by terrain and other conditions, the actual regulation and storage volume is small
Biological retention facility	Various forms, wide application area, easy to integrate with the landscape, good runoff control effect, low construction and maintenance costs	In areas with high groundwater levels and rock layers, poor soil permeability, and steep terrain, necessary measures such as soil replacement, seepage prevention, and ladder installation should be taken to avoid secondary disasters, which will increase construction costs.
Permeation pond	Can effectively supplement groundwater, reduce peak flow, and lower construction costs	Strict requirements for site conditions and high requirements for later maintenance and management
Seepage well	Small footprint, low construction and maintenance costs	The water quality and quantity control effects are limited
Wet pond	It can effectively reduce the total amount of runoff, runoff pollution, and peak flow in a larger area	Strict requirements for on-site conditions, high construction and maintenance costs
Rainwater wetland	Can effectively reduce pollutants, has a certain runoff and peak flow control effect	Higher construction and maintenance costs
Reservoir	It has the advantages of saving land, easy access to rainwater pipes, avoiding direct sunlight, preventing mosquitoes and flies, and storing large amounts of water. Rainwater can be reused for green irrigation, washing roads and vehicles, etc.	The construction cost is high, and maintenance and management should be paid attention in the later period
Rainwater tank	Mostly molded products, convenient for construction and installation, and easy for maintenance	The storage volume is small, and rainwater purification capacity is limited
Regulating pond	Can effectively reduce peak traffic, lower construction and maintenance costs	The function is relatively simple
Regulating pool	Can effectively reduce peak traffic	The function is simple, high construction and maintenance costs
Grassed swales	Low construction and maintenance costs, easy to integrate with the landscape	Areas such as built urban areas and newly built urban areas with greater development intensity are vulnerable to site conditions
Seepage pipe/drain	Small space requirements for the site	The construction cost is high, it gets blocked easily, and is difficult to maintain
Vegetation buffer zone	Low construction and maintenance costs	High requirements for site space, slope, and other conditions, and limited runoff control effects
Initial rainwater discarding facility	Small footprint and low construction costs, which can reduce the maintenance and management costs of rainwater storage and rainwater purification facilities	Runoff pollutants and discarded flow are generally not easy to control
Artificial soil infiltration	Infiltration rainwater purification effect is good, easy to integrate with the landscape	High construction costs

The article "The Control Index for the Construction of Sponge City in the Residential Area: A Case Study of Nanjing Jiangbei New District" was published in 2022. Journal: J Environ Public Health.

**Table 9:** Comparison of low-impact development facilities.

Single facility	Functions					Control objectives			Solving method		Economy	Economy	Pollutant removal rate (calculated by SS,%)	Landscape effect
	Collecting and storing rainwater	Supplementing groundwater	Reducing peak flow	Purifying rainwater	Transmission	Total runoff	Peak runoff	Runoff pollution	Dispersion	Relatively concentrated	Construction costs	Maintenance costs		
Permeable brick paving	○	●	◎	◎	○	●	◎	◎	√	-	Low	Low	80-90	-
Permeable cement concrete	○	○	◎	◎	○	◎	◎	◎	√	-	High	Medium	80-90	-
Permeable asphalt concrete	○	○	◎	◎	○	◎	◎	◎	√	-	High	Medium	80-90	-
Green roof	○	○	◎	◎	○	●	◎	◎	√	-	High	Medium	70-80	Good
Sunken green space	○	●	◎	◎	○	●	◎	◎	√	-	Low	Low	-	Fair
Simple biological retention facility	○	●	◎	◎	○	●	◎	◎	√	-	Low	Low	-	Good
Complex biological retention facility	○	●	◎	●	○	●	◎	●	√	-	Medium	Low	70-95	Good
Permeation pond	○	●	◎	◎	○	●	◎	◎	-	√	Medium	Medium	70-80	Fair
Seepage well	○	●	◎	◎	○	●	◎	◎	√	√	Low	Low	-	-
Wet pond	●	○	●	◎	○	●	●	◎	-	√	High	Medium	50-80	Good
Rain wetland	●	○	●	●	○	●	●	●	√	√	High	Medium	50-80	Good
Reservoir	●	○	◎	◎	○	●	◎	◎	-	√	High	Medium	80-90	-
Rainwater tank	●	○	◎	◎	○	●	◎	◎	√	-	Low	Low	80-90	-
Regulating pond	○	○	●	◎	○	●	●	◎	-	√	High	Medium	-	Fair
Regulation pool	○	○	●	○	○	●	●	○	-	√	High	Medium	-	-
Transmission type grassed swales	◎	○	○	◎	●	○	○	◎	√	-	Low	Low	35-90	Fair
Dry grassed swales	○	●	○	◎	●	○	○	◎	√	-	Low	Low	35-90	Good
Wet grassed swales	○	○	○	●	●	◎	○	●	√	-	Medium	Low	-	Good
Seepage pipe/drain	○	◎	○	○	●	●	○	◎	√	-	Medium	Medium	35-70	-
Vegetation buffer zone	○	○	○	●	-	○	○	●	√	-	Low	Low	50-75	Fair
Initial rainwater discarding facility	◎	○	○	●	-	○	○	●	√	-	Low	Medium	40-60	-
Artificial soil infiltration	●	○	○	●	-	○	○	◎	-	√	High	Medium	75-95	Good

*Note.* ●-Strong ◎-Relatively strong ○-Weak or very small; The 2SS removal rate data come from the research data of the Center for Watershed Protection (CWP) of the United States.

## Data Availability

The data used to support the findings of this study are included within the article.
